The article "HMGB1 regulates SNAI1 during NSCLC metastasis, both directly, through transcriptional activation, and indirectly, in a RSF1‐IT2‐dependent manner" was retracted in 2022. Reasons: duplicated images; unreliable results or conclusions; concerns about the data.

# HMGB1 regulates SNAI1 during NSCLC metastasis, both directly, through transcriptional activation, and indirectly, in a RSF1‐IT2‐dependent manner

**DOI:** 10.1002/1878-0261.12691

**Published:** 2020-05-06

**Authors:** Xiao‐jin Wu, Yuan‐yuan Chen, Wen‐wen Guo, Tao Li, Hai‐bei Dong, Wei Wang, Min Xie, Gao‐lei Ma, Dong‐sheng Pei

**Affiliations:** ^1^ Department of Radiation Oncology The Affiliated Xuzhou Municipal Hospital of Xuzhou Medical University Xuzhou First People's Hospital China; ^2^ Department of Respiratory The Affiliated Xuzhou Municipal Hospital of Xuzhou Medical University Xuzhou First People's Hospital China; ^3^ Department of Pathology Xuzhou Medical University China

**Keywords:** HMGB1, miR‐129‐5p, NSCLC, RSF1‐IT2, SNAI1

## Abstract

High‐mobility group protein B1 (HMGB1) has important functions in cancer cell proliferation and metastasis. However, the mechanisms of HMGB1 function in non‐small‐cell lung cancer (NSCLC) remain unclear. This study aimed to investigate the underlying mechanism of HMGB1‐dependent tumor cell proliferation and NSCLC metastasis. Firstly, we found high HMGB1 expression in NSCLC and showed that HMBG1 promoted proliferation, migration, and invasion of NSCLC cells. HMGB1 could bind to SNAI1 promoter and activate the expression of SNAI1. In addition, HMGB1 could transcriptionally regulate the lncRNA RSF1‐IT2. RSF1‐IT2 was found to function as ceRNA, sponging miR‐129‐5p, which targets SNAI1. Notably, HMGB1 was also identified as a target of miR‐129‐5p, which indicates the establishment of a positive feedback loop. Consequently, high expression of RSF1‐IT2 and SNAI1 was found to closely correlate with tumor progression in both HMGB1‐overexpressing xenograft nude mice and patients with NSCLC. Taken together, our findings provide new insights into molecular mechanisms of HMGB1‐dependent tumor metastasis. Components of the HMGB1–RSF1‐IT2–miR‐129‐5p–SNAI1 pathway may have a potential as prognostic and therapeutic targets in NSCLC.

## Graphical abstract

Dual‐mode regulation of SNAI1 by HMGB1 in NSCLC metastasis.

**Abbreviations**
CCK‐8: Cell Counting Kit‐8
EMT: epithelial–mesenchymal transition
HMGB1: high‐mobility group protein B1
IRS: immunoreactive score
lncRNA: long noncoding RNA
NSCLC: non‐small‐cell lung cancer
NTs: noncancerous tissues
RAGE: receptor for advanced glycation end products
RSF1‐IT2: remodeling and spacing factor 1‐intronic transcript 2
TLR: toll‐like receptor

## 1 Introduction

Lung cancer is the most common malignant tumor with high morbidity and mortality worldwide, 80–85% of which is pathologically diagnosed with non‐small‐cell lung cancer (NSCLC) including squamous cell carcinoma, adenocarcinoma, and large cell carcinoma (Asamura *et al.*, 2015; Ettinger *et al.*, 2016). Although there are diverse treatments for NSCLC such as surgery, radiotherapy, chemotherapy, and targeted therapy, the overall 5‐year survival rate is only 18.2% (Feng *et al.*, 2016). Tumor metastasis is the leading cause of death in NSCLC patients, and it is regulated by many complex factors (Borghaei *et al.*, 2015). Therefore, exploring the molecular mechanism of NSCLC metastasis is conducive to find efficient strategies to inhibit tumor growth and improve the therapeutic effect.

High‐mobility group protein B1 (HMGB1), a ubiquitous nuclear protein, plays a significant role in regulating transcription, replication, repair, and genetic stability (Wu *et al.*, 2018b; Wu and Yang, 2018). Intracellular HMGB1 mainly acts in the nucleus and regulates gene expression as an architectural chromatin‐binding protein, while extracellular HMGB1 can bind receptor for advanced glycation end products (RAGE) and toll‐like receptor (TLR) inducing multiple biological effects (Luan *et al.*, 2018). Recent studies have shown that HMGB1 is highly expressed in various human carcinomas (Chuangui *et al.*, 2012; Wu and Yang, 2018). Moreover, high HMGB1 expression is significantly associated with advanced stages, distant metastasis, and poor prognosis in lung cancer patients (Liu *et al.*, 2017; Postmus *et al.*, 2013; Wu *et al.*, 2018a). It is indicated that HMGB1 can act as an effective therapeutic target to offer a new way for the treatment of lung cancer.

Long noncoding RNAs (lncRNAs) are a class of non‐protein coding transcripts with a length greater than 200 nucleotides. Recently, lncRNAs have attracted more attention because of its important role in transcription, translation, epigenetic modification, and cell cycle regulation (Xuan *et al.*, 2019; Yao and Wang, 2019). Emerging evidence revealed that lncRNAs were abnormally expressed in various cancer types and affected tumor metastasis (Yao and Wang, 2019). Remodeling and spacing factor 1 (RSF1), which is one of chromatin‐remodeling factors, has been demonstrated to be highly expressed and associated with poor prognosis in NSCLC, renal cancer, and ovarian cancer (Wu *et al.*, 2017; Yang *et al.*, 2014; Zhang *et al.*, 2018). RSF1‐intronic transcript 2 (RSF1‐IT2), derived from an intron within the RSF1 gene, has been mapped to chromosome 11 region 77717712–77718741 reverse strand according to the NCBI. RSF1‐IT2 was located in 11q14 with 2 exons, and its role in cancers remained largely unknown.

Previous studies have shown that HMGB1 accelerates tumor growth and metastasis (Chuangui *et al.*, 2012; Lv *et al.*, 2016; Wang *et al.*, 2015). However, the molecular mechanisms and downstream effector pathways of HMGB1 in NSCLC are still unclear. Moreover, the role of RSF1‐IT2 in cancers and the mechanism of its regulation by HMGB1 have not been reported. The present study focused on the investigation of HMGB1‐induced tumor metastasis and regulated RSF1‐IT2, hoping to further clarify the signaling pathway of HMGB1 and provide novel therapeutic target for the treatment of NSCLC.

## 2 Materials and methods

### 2.1 Tissue samples and cell lines

The tissue specimens were consisted of 122 NSCLC tissues and 120 noncancerous tissues (NTs). All patients were primary pathologically diagnosed with NSCLC at Affiliated Xuzhou Municipal Hospital of Xuzhou Medical University between July 2007 and June 2011, and followed up for 5 years. The study methodologies conformed to the standards set by the Declaration of Helsinki.

H1299 and H460 cells were obtained from the American Type Culture Collection (ATCC, Manassas, VA, USA). H1299 and H460 cells were cultured in Roswell Park Memorial Institute 1640 medium supplemented with 10% bovine blood serum (Sijiqing Laboratories, Hangzhou, Zhejiang, China) at 37 °C in a humidified atmosphere with 5% CO_2_.

### 2.2 Transfection

siRNAs were purchased from GenePharma, Shanghai, China. The sequences of all oligos used for transfections were as follows: of si‐HMGB1, sense, 5′‐GCAUAAGAAGAAGCACCCATT‐3′, of si‐SNAI1, sense, 5′‐GGCCUUCAACUGCAAAUAUTT‐3′, of si‐RSF1‐IT2, sense, 5′‐CAAGCTTTGATATTTTAAGGAGATTCATTTTTG‐3′. The cells were transfected with siRNA using siLentFect Lipid Reagent (Bio‐Rad, Hercules, CA, USA). The pcDNA3.1, pcDNA3.1‐HMGB1 plasmids, and pcDNA3.1‐RSF1‐IT2 plasmids were purchased from Guangzhou FulenGen Co. (Guangzhou, Guangdong, China), which were transfected using X‐tremeGENE HP DNA Transfection Reagent (Roche, Indianapolis, IN, USA). The LV‐Vector‐H1299 and LV‐HMGB1‐H1299 cells were established by infected with lentiviruses (GenePharma).

### 2.3 Transwell assay

Migration or invasion assays were performed with the transwell inserts (Corning Incorporated, New York, NY, USA) with or without Matrigel (BD Biosciences, San Jose, CA, USA). Cells were immobilized for 15 min with 4% paraformaldehyde (Vicmed, Xuzhou, China) and stained with crystal violet staining (Vicmed). The results were taken with Nikon digital camera (Pan *et al.*, 2017).

### 2.4 Wound healing assay

After transfection, H1299 and H460 cells pretreated with mitomycin C (10 µg·mL^−1^) were harvested and seeded into 6‐well plates. A linear scratch/wound was created on cell monolayers using a pipette tip. Photomicrographs were taken of live cells at ×100 magnification with a Nikon digital camera (Nikon, Toyko, Japan), and the distance migrated was observed within an appropriate time.

### 2.5 Cell proliferation assay

After transfection, H1299 and H460 cells (4 × 10^3^) were cultured in 96‐well microplate (Corning Incorporated) in triplicate. Then, 10 µL Cell Counting Kit‐8 (CCK‐8; Vicmed) solution was added to each well at 24, 48, 72, and 96 h, respectively. Absorbance was measured at 450 nm by a multifunctional enzyme‐linked analyzer (BioTek Instruments, Winooski, VT, USA).

### 2.6 EdU staining

H1299 and H460 cells were cultured in 24‐well plate and transfected with si‐HMGB1 or pcDNA3.1‐HMGB1. After transfection, the cells were incubated with 3.7% neutral methanol for 15 min, and then 0.1% Triton X‐100 for 15 min and 10 μm EdU for 30 min using keyFlour488 Click‐It EdU imaging detection kit (KeyGEN Biotech, Nanjing, China). The results were captured with a Nikon fluorescence inversion microscope (Pan *et al.*, 2017).

### 2.7 Cell apoptosis assay

After transfection, cells were washed twice with ice‐cold PBS, then incubated with 200 µL 1 × binding buffer containing 5 µL Annexin V‐FITC, and then with 300 µL 1 × binding buffer containing 5 µL propidium iodide (PI) for 10 min at room temperature in the dark using the Annexin V‐FITC Kit (FITC Annexin V Apoptosis Detection Kit I; BD). After incubation, cells were visualized under a fluorescence microscope.

### 2.8 Immunohistochemistry and RNAscope

Tissues were cut into 4‐mm sections, and then deparaffinized and rehydrated. Endogenous peroxidase activity was blocked with 0.3% hydrogen peroxide for 15 min. After blocking with 5% normal goat serum for 30 min, slides were incubated with the primary antibodies overnight at 4 °C followed by secondary antibody for 15 min. The slides were then counterstained with hematoxylin. The staining intensity was scored 0–3 (0 = negative; 1 = weak; 2 = moderate; 3 = strong). The percentage of positive stained cells was scored 0–4: 0 (0%), 1 (1–25%), 2 (26–50%), 3 (51–75%), or 4 (76–100%). The immunoreactive score (IRS) was calculated by multiplying the scores of staining intensity and the percentage of positive cells. IRS of 0–1 was defined as low expression, and IRS of 2–12 was defined as high expression (Lv *et al.*, 2019).

The RNAscope probe was designed and synthesized by Advanced Cell Diagnostics Company (Newark, CA, USA). RSF1‐IT2 and miR‐129‐5p expression were detected using an RNAscope 2.5 High Definition (HD)‐BROWN Assay Kit (Advanced Cell Diagnostics). The signals were scored based on the average number of dots per cell: 0 (0–1 dots/10 cells), 1 (1–3 dots/cell), 2 (4–10 dots/ cell), 3 (> 10 dots/cell with dots in clusters), and 4 (> 15 dots/cell and > 10% of the dots presented in clusters). Based on the scores, staining pattern was defined as low (score: 0–1) and high (score: 2–4) (Jin *et al.*, 2019).

### 2.9 Western blot

After performing specific treatments, cells were washed with ice‐cold PBS twice and lysed in lysis buffer (Beyotime, Shanghai, China). Proteins were separated on SDS/PAGE and transferred to nitrocellulose filter membrane. Membranes were incubated in turn with 5% bovine serum for 2 h, primary antibody overnight at 4 °C, and secondary antibody for 2 h. The densities of the bands on the membrane were scanned and analyzed with imagej (LabWorks Software, UVP Upland, CA, USA) (Zhang *et al.*, 2017).

### 2.10 Luciferase reporter assay

Cells were split into 48‐well plates, and each well was transfected with plasmids following the manufacturer's procedures. After 24 h, whole‐cell lysate was collected and their luciferase activities were evaluated using Dual‐Luciferase Kit (Promega, Shanghai, China). Reactions were measured using an Orion Microplate Luminometer (Berthold Detection System, Bad Wildbad, Germany).

### 2.11 Chromatin immunoprecipitation assay

The EZ ChIP kit (Upstate, NY, USA) was used. Firstly, the cells are treated with ultrasound to disrupt chromatin DNA fragments in the cells to 200–500 bp. The sonicated cells were centrifuged, and the supernatants were aspirated. The supernatants were inverted with anti‐HMGB1 or normal rabbit IgG at 4 °C overnight. The cross‐linked DNA‐protein was heated at 65 °C overnight and then subjected to PCR analysis (Zuo *et al.*, 2014).

### 2.12 Quantitative real‐time RT‐PCR

Total RNA from H1299 and H460 cells was extracted using TRIzol reagent and used as a template for cDNA synthesis. Lnc RNAs, miRNAs, and mRNAs were reverse‐transcribed by using PrimeScript RT Master Mix (Takara, Dalian, China). RT‐PCR was performed with ABI StepOne (Carlsbad, CA, USA) following the instructions. The relative quantification of miR‐129‐5p was carried out by the $2^{-\Delta \Delta C_{T}}$ method, where U6 was used as the control gene. The expression levels of HMGB1, RSF1‐IT2, and SNAI1 were normalized to the levels of internal control GAPDH. Primers for the individual genes were as follows: GAPDH forward, 5′‐CAAGGTCATCCATGACAACTTTG‐3′; GAPDH reverse, 5′‐GTCCACCACCCTGTTGCTGTAG‐3′; U6 forward, 5′‐GCTTCGGCAGCACATATACTAAAAT‐3′; U6 reverse, 5′‐CGCTTCACGAATTTGCGTGTCAT‐3′; HMGB1 forward, 5′‐ATGCTTCAGTCAACTTCTCAGA‐3′; HMGB1 reverse, 5′‐CATTTCTCTTTCATAACGGGCC‐3′; RSF1‐IT2 forward, 5′‐CCAGGCTGGAGCACAATGGC‐3′; RSF1‐IT2 reverse, 5′‐AGGCTGAGGCAGGAGAATCGG‐3′; miR‐129‐5p forward, 5′‐CGCTTTTTGCGGTCTGG‐3′; miR‐129‐5p reverse, 5′‐AGTGCAGGGTCCGAGGTATT‐3′; SNAI1 forward, 5′‐GGCTCCTTCGTCCTTCTCCTCTAC‐3′; SNAI1 reverse, 5′‐CCAGGCTGAGGTATTCCTTGTTGC‐3′.

### 2.13 Bioinformatics analysis

Firstly, mircode (http://www.mircode.org/) website was used for prediction of lncRNA and miRNA targets. Then, miRNA‐mRNA pairs were established using online analysis tools, namely TargetScan (http://www.targetscan.org) and mircode (http://www.mircode.org/).

### 2.14 Xenograft tumor model in nude mice

Four‐ to five‐week‐old female BALB/c nude mice were purchased from Shanghai Experimental Animal Center of Chinese Academy of Sciences (Shanghai, China) and quarantined for a week before tumor implantation. The NSCLC xenograft model was established by tail intravenous injection of 2 × 10^6^ H1299 cells (transfected with LV‐Vector or LV‐HMGB1). The mice were put to death after 4 weeks of rearing (*n* = 12 for each group). Lungs were surgically retrieved from mice, and tumor nodules at lung surface were counted.

### 2.15 Statistical analysis

Two‐tailed Student's *t*‐test was performed to calculate significance in an interval of 95% confidence level. Statistical differences between the means for the different groups were evaluated with instat 5.0 (GraphPad Software, San Diego, CA, USA) using one‐way analysis of variance (ANOVA). The Pearson correlation coefficient was used for correlation analysis. All values are shown as mean ± SD, and a value of *P* < 0.05 was considered statistically significant. The association between HMGB1 staining and the clinicopathological parameters of the NSCLC patients, including ages, pT status, pN status, and TNM stage, was evaluated by chi‐square test. The Kaplan–Meier method and log‐rank test were used to evaluate the correlation between HMGB1 expression and patient survival.

## 3 Results

### 3.1 HMGB1 expression is high in NSCLC tissues and serves as a potential prognostic indicator for NSCLC

We firstly detected the expression levels of HMGB1 by immunohistochemistry in tissue microarray slides containing 122 NSCLC tissues and 120 paired adjacent NTs. NSCLC tissues exhibited various degrees of HMGB1 expression (Fig. 1A). High HMGB1 expression staining was observed in 82 of 122 (67.4%) NSCLC tissues and 10 of 122 (8.3%) adjacent NTs. Increasing HMGB1 expression was significantly correlated with advanced TNM stages (*P* = 0.000) and metastasis (*P* = 0.026). However, we did not find a significant association of HMGB1 expression with patient's age or sex (Fig. 1B,C). Through Kaplan–Meier and log‐rank test analyses in 122 NSCLC patients, high HMGB1 expression was correlated with worse overall survival time (*P* < 0.05, Fig. 1D). Furthermore, we found that TNM stage (I–II vs III–IV, *P* = 0.001), pT status (T1‐2 vs T3‐4, *P* = 0.001), pN status (N0 vs N+, *P* = 0.022), and HMGB1 staining (− vs +, *P* = 0.023) were the risk factors for death in NSCLC patients (Table. 1), wherein that TNM stage (*P* = 0.0014), pT status (*P* = 0.005) and pN status (*P* = 0.001) were the independent risk factors for death in NSCLC patients by using Cox multivariate regression analysis (Table 2).

**Fig. 1:** HMGB1 expression is high in NSCLC tissues and serves as a potential prognostic indicator for NSCLC. (A) Representative images of HMGB1 immunohistochemical staining in NSCLC patients. Magnification ×100, ×200, ×400. (B, C) Association between HMGB1 expression and clinicopathological features in NSCLC tissues (*P < 0.05, **P < 0.01, ***P < 0.001, NS, no significance, χ^2^ test). (D) High HMGB1 expression correlated with worse overall survival over a 5‐year period in 122 NSCLC patients (HMGB1^High^ *n* = 82, HMGB1^Low^ *n* = 40, *P* < 0.05, log‐rank test).

**Table 1:** Cox univariate regression analysis of the risk factors for death in lung cancer patients.

Pathology character	HR	95% CI	*P* value
Age (year)	1.555	0.896–2.696	0.116
Gender	0.545	0.31–0.957	0.035*
TNM stage (I–II vs III–IV)	1.506	1.199–1.892	0.000*
pT status (T1‐2 vs T3‐4)	3.892	1.806–8.386	0.001*
pN status (N0 vs N+)	1.042	0.736–1.474	0.818
Metastasis (M0 vs M1)	2.054	0.492–8.570	0.324
HMGB1 staining (− vs +)	1.996	1.058–3.766	0.033*

*P < 0.05.

**Table 2:** Cox multivariate regression analysis of independent risk factors for death in lung cancer patients.

Pathology character	HR	95% CI	*P* value
Gender	0.466	0.257–0.844	0.012*
TNM stage (I–II vs III–IV)	4.388	1.367–14.084	0.967
pT status (T1‐2 vs T3‐4)	2.919	1.026–8.305	0.045*
HMGB1 staining (− vs +)	2.143	1.074–4.274	0.031*

*P < 0.05.

### 3.2 HMGB1 promotes NSCLC invasion and migration through the up‐regulation of SNAI1 expression

Next, we performed loss‐of‐function and gain‐of‐function experiments to explore the biological role of HMGB1 in NSCLC cells. The results indicated that HMGB1 accelerated tumor proliferation and inhibited apoptosis in NSCLC cells (Fig. 2A–D). After that, we observed that HMGB1 remarkably promoted cell migration and invasion in H1299 and H460 cells (Fig. 2E,F). To figure out the mechanism of HMGB1 promoting metastasis, the expression of the epithelial–mesenchymal transition (EMT) markers was analyzed by western blot. It revealed that SNAI1, Twist, and Vimentin were significantly increased after overexpressing HMGB1 and attenuated after silencing HMGB1 (Fig. 2G). Moreover, cotransfection of the SNAI1 promoter with HMGB1 plasmid resulted in multiplied promoter activity and HMGB1 could directly bind the SNAI1 promoter region (Fig. 2H,I). Besides, SNAI1 knockdown could reverse the induction of tumor invasion by HMGB1 in NSCLC cells (Fig. 2J). These results manifested that HMGB1 promoted NSCLC migration and invasion through up‐regulating SNAI1 expression at the transcriptional level.

**Fig. 2:** HMGB1 promotes NSCLC invasion and migration through the up‐regulation of SNAI1 expression. (A) Representative images of EdU staining after transfection of siHMGB1 or pcDNA3.1‐HMGB1. The EdU‐positive cells were measured and shown as a bar graph (scale bar, 100 μm). (B) The cell proliferation was detected by CCK‐8 assays after transfection of siHMGB1 or pcDNA3.1‐HMGB1, at 24, 48, and 72 h. (C) Western blot analysis of HMGB1, cleaved caspase‐3, cleaved PARP in H1299 and H460 cells after transfection with siHMGB1 or pcDNA3.1‐HMGB1. (D) Annexin V‐FITC binding assay was used to observe apoptotic cells by fluorescence microscope in NSCLC cells transfected with siHMGB1 or pcDNA3.1‐HMGB1 and their negative control (scale bar, 100 μm). (E) Representative images of the wound healing distance of shift after transfection with siHMGB1 or pcDNA3.1‐HMGB1 in H1299 and H460 cells. (F) The cell migration and invasion of H1299 and H460 cells after transfection with siHMGB1 or pcDNA3.1‐HMGB1 were detected by transwell assays. (G) Western blot analysis of HMGB1, Twist, SNAI1, Vimentin, β‐catenin, N‐cadherin, E‐cadherin, and Fibronectin in H1299 and H460 cells after transfection with siHMGB1 or pcDNA3.1‐HMGB1. (H) Luciferase reporter assay was carried out in H1299 and H460 cells. The relative luciferase activities of cotransfection of the SNAI1, Twist, and Vimentin with HMGB1 plasmid against pcDNA3.1(+)+pGL3‐SNAI1, pcDNA3.1(+)+pGL3‐Twist, and pcDNA3.1(+)+pGL3‐Vimentin group. (I) Soluble chromatins of H1299 and H460 cells were prepared and subjected to ChIP assay using anti‐HMGB1 antibody as described in the section of ‘Materials and methods’. (J) The cell migration and invasion of LV‐Vector‐H1299 and LV‐HMGB1‐H1299 cells after transfection with siNC and si‐SNAI1 were detected by transwell assays. All experiments were performed three times (*n* = 3, the data were presented as mean ± SD. Student's *t*‐test was used to determine statistical significance: *P < 0.05, **P < 0.01, ***P < 0.001).

### 3.3 HMGB1‐induced RSF1‐IT2 promotes NSCLC cell migration and invasion through sponging miR‐129‐5p

As a nonhistone DNA‐binding protein, HMGB1 could affect lncRNA expression in lung cancer progression. Therefore, we selected the top 30 up‐regulated lncRNAs in NSCLC using TCGA database and performed qPCR to ulteriorly verify whether HMGB1 regulated lncRNA level in cancer metastasis (Figs S1 and S2). Intriguingly, it was found that HMGB1 could increase the expression of RSF1‐IT2 through binding RSF1‐IT2 promoter (Fig. 3A,B, Fig. S3). Thus, we inferred that RSF1‐IT2 could function as an oncogene to accelerate NSCLC cell proliferation and invasion. It was indicated that RSF1‐IT2 overexpression was effective in promoting NSCLC cell growth and invasiveness (Fig. 3C,D). In the meantime, RSF1‐IT2 increased SNAI1 expression at the levels of RNA and protein (Fig. 3E,F). To certify the mechanism of RSF1‐IT2 promoting cell invasion, we used mircode (http://www.mircode.org/) software to search for the predicted potential target miRNAs of RSF1‐IT2. The data revealed that miR‐129‐5p had putative RSF1‐IT2 binding sites and was down‐regulated by RSF1‐IT2, indicating RSF1‐IT2 could act as a ceRNA for miR‐129‐5p thus facilitating metastasis in NSCLC (Fig. 3G,H, Fig. S4). Furthermore, miR‐129‐5p mimics attenuated the effect of RSF1‐IT2 on tumor growth and invasion (Fig. 3I,J). Together with these observations, RSF1‐IT2 induced NSCLC cell proliferation, migration, and invasion through sponging miR‐129‐5p.

**Fig. 3:** HMGB1‐induced RSF1‐IT2 promotes NSCLC cell migration and invasion through sponging miR‐129‐5p. (A) H1299 and H460 cells were transfected with si‐HMGB1 and pcDNA3.1‐HMGB1. qPCR showed that pcDNA3.1‐HMGB1 up‐regulated RSF1‐IT2 expression and si‐HMGB1 decreased RSF1‐IT2 expression. (B) The effect of si‐HMGB1 or pcDNA3.1‐HMGB1 on promoter activity of RSF1‐IT2 was compared via luciferase reporter assay in H1299 cells. (C) Effects of RSF1‐IT2 on the growth of H1299 and H460 cells. (D) RSF1‐IT2 promoted NSCLC cell invasion and migration, as measured by transwell assay. (E) qPCR showed that pcDNA3.1‐RSF1‐IT2 up‐regulated SNAI1 expression and si‐RSF1‐IT2 decreased SNAI1 expression. (F) Western blot showed that SNAI1 expression increased in pcDNA3.1‐RSF1‐IT2 group and decreased in si‐RSF1‐IT2 group. β‐actin is the internal control. (G) After transfected with si‐RSF1‐IT2 and pcDNA3.1‐RSF1‐IT2, qPCR showed that pcDNA3.1‐RSF1‐IT2 decreased miR‐129‐5p expression and si‐RSF1‐IT2 increased miR‐129‐5p expression. (H) WT‐RSF1‐IT2 or MUT‐RSF1‐IT2 was cotransfected into H1299 cells with miR‐129‐5p mimics or their corresponding negative controls. (I) CCK‐8 assay showed that miR‐129‐5p mimics attenuated the proliferation‐promoting effect of RSF1‐IT2 in H1299 and H460 cells. (J) miR‐129‐5p mimics attenuated the effect of RSF1‐IT2 on cell invasion and migration, as measured by transwell assay. All experiments were performed three times (*n* = 3, the data were presented as mean ± SD. Student's *t*‐test was used to determine statistical significance: *P < 0.05, **P < 0.01, ***P < 0.001; NS, no significance).

### 3.4 MiR‐129‐5p targets both SNAI1 and HMGB1

Since RSF1‐IT2 can sponge miR‐129‐5p, the interactions between miR‐129‐5p and SNAI1 were explored. After being treated with miR‐129‐5p mimics, SNAI1 expression was evidently reduced, and knockdown of miR‐129‐5p up‐regulated SNAI1 (Fig. 4A,B). Through blasting the binding site of miR‐129‐5p and SNAI1, we constructed luciferase vectors of mutant SNAI1 3′UTR and wild‐type. The results proved that the luciferase activities were significantly decreased after transfected with wild‐type SNAI1 3′UTR vector together with miR‐129‐5p mimics, but not mutant SNAI1 3′UTR (Fig. 4C,D). Interestingly, we found miR‐129‐5p also targeted HMGB1 through mircode (http://www.mircode.org/) software. Similarly, miR‐129‐5p could inhibit the expression of HMGB1 (Fig. 4E,F). The luciferase activity reflected the interaction between wild‐type HMGB1 3′UTR and miR‐129‐5p mimics (Fig. 4G,H). In a word, the above data demonstrated the negative regulatory effect of miR‐129‐5p on SNAI1 and HMGB1 expression.

**Fig. 4:** MiR‐129‐5p targets both SNAI1 and HMGB1. (A) qRT‐PCR showed that miR‐129‐5p inhibitor up‐regulated SNAI1 expression and miR‐129‐5p mimics decreased SNAI1 expression (*n* = 3, mean ± SD, *t*‐test). (B) Western blot showed SNAI1 increased in miR‐129‐5p inhibitor group and decreased in miR‐129‐5p mimics group in H1299 and H460 cells. β‐actin is the internal control. (C) The potential binding sites between SNAI1 and miR‐129‐5p. (D) WT‐SNAI1 or MUT‐SNAI1 was cotransfected into H1299 cells with miR‐129‐5p mimics or their corresponding negative controls (*n* = 3, mean ± SD, *t*‐test). (E) qPCR showed that miR‐129‐5p inhibitor up‐regulated HMGB1 expression and miR‐129‐5p mimics decrease HMGB1 expression (*n* = 3, mean ± SD, *t*‐test). (F) Western blot showed HMGB1 increased in miR‐129‐5p inhibitor group and decreased in miR‐129‐5p mimics group in H1299 and H460 cells. β‐actin was the internal control. (G) The potential binding sites between HMGB1 and miR‐129‐5p. (H) WT‐HMGB1 or MUT‐HMGB1 was cotransfected into H1299 cells with miR‐129‐5p mimics or their corresponding negative controls (*n* = 3, mean ± SD, *t*‐test) (*P < 0.05, **P < 0.01, ***P < 0.001).

### 3.5 RSF1‐IT2 and SNAI1 are up‐regulated, whereas miR‐129‐5p is down‐regulated in NSCLC tissues

Next, we investigated RSF1‐IT2, SNAI1, and miR‐129‐5p expression in 122 NSCLC tissues. RSF1‐IT2 high expression was observed in 49 of 82 (59.8%) HMGB1 highly expressed NSCLC tissues (Fig. 5A,B). RSF1‐IT2 expression was elevated in NSCLC tissues, and high RSF1‐IT2 expression was associated with advanced TNM stages, metastasis, and poor prognosis (Fig. 5C,D). SNAI1 was also expressed in different levels through immunohistochemistry in 122 NSCLC tissues. SNAI1 expression was positively correlated with HMGB1 expression (Fig. 5E,F). Meanwhile, SNAI1 high expression was related to advanced TNM stages, metastasis, and poor prognosis in NSCLC (Fig. 5G,H). Additionally, miR‐129‐5p was negatively correlated with HMGB1 expression and down‐regulated in most NSCLC tissues compared with adjacent NTs (Fig. 5I–K). The reduced expression of miR‐129‐5p was linked with advanced TNM stages, metastasis, and poor prognosis (Fig. 5K,L).

**Fig. 5:** RSF1‐IT2 and SNAI1 are up‐regulated, whereas miR‐129‐5p is down‐regulated in NSCLC tissues. (A) Representative images of RSF1‐IT2 staining in NSCLC tissues (scale bar, 100 μm). (B) High RSF1‐IT2 expression was correlated with high HMGB1 expression. (C) Association between RSF1‐IT2 expression and clinical–pathological features in NSCLC tissues (*P < 0.05, **P < 0.01, ***P < 0.001, χ^2^ test). (D) High RSF1‐IT2 expression was correlated with a worse 5‐year overall cumulative survival for 122 NSCLC patients (RSF1‐IT2^High^ *n* = 63, RSF1‐IT2^Low^ *n* = 59, *P* < 0.05, log‐rank test). (E) Representative images of SNAI1 staining in NSCLC tissues (scale bar, 100 μm). (F) High SNAI1 expression was correlated with high HMGB1 expression. (G) Association between SNAI1 expression and clinical–pathological features in NSCLC tissues (*P < 0.05, **P < 0.01, ***P < 0.001, χ^2^ test). (H) High SNAI1 expression was correlated with a worse 5‐year overall cumulative survival for 122 NSCLC patients (SNAI1^High^ *n* = 75, SNAI1^Low^ *n* = 47, *P* < 0.05, log‐rank test). (I) Representative images of miR‐129‐5p staining in NSCLC tissues (scale bar, 100 μm). (J) Low miR‐129‐5P expression was correlated with high HMGB1 expression. (K) Association between miR‐129‐5p expression and clinical–pathological features in NSCLC tissues (*P < 0.05, **P < 0.01, ***P < 0.001, χ^2^ test). (L) Low miR‐129‐5p expression was correlated with worse overall survival over a 5‐year period for 122 NSCLC patients (miR‐129‐5p^High^ *n* = 53, miR‐129‐5p^Low^ *n* = 69, *P* < 0.05, log‐rank test).

### 3.6 HMGB1 promotes RSF1‐IT2 and SNAI1 expression, as well as NSCLC metastasis *in vivo*

To investigate the effect of HMGB1 on NSCLC metastasis *in vivo*, xenograft cancer models were established by subcutaneously inoculating H1299 cells stably transfected with HMGB1 (Fig. 6A). Through observation, it was found that the mice injected with LV‐HMGB1‐H1299 cells exhibited more metastatic nodules (*P* < 0.001, Fig. 6B). Pathological report of lung nodules was consistent with metastatic tumor of NSCLC (Fig. 6C). Additionally, we observed that RSF1‐IT2 and SNAI1 expression increased, whereas miR‐129‐5p expression decreased from harvested tumor tissues in the LV‐HMGB1 group (Fig. 6D–F). These findings were identical to the *in vitro* results described above, which firmly validated that HMGB1 promoted RSF1‐IT2 and SNAI1 expression as well as NSCLC metastasis *in vivo*.

**Fig. 6:** HMGB1 promotes expression of RSF1‐IT2 and SNAI1, as well as NSCLC metastasis *in vivo*. (A) Fluorescence microscope and western blot detect the infection efficiency of lentivirus in H1299 cells (magnification ×100, scale bar 100 μm). (B) Representative images of lungs with metastatic nodules 4 weeks after injection of LV‐Vector‐H1299 or LV‐HMGB1‐H1299 cells (*n* = 12, mean ± SD, *t*‐test, ***P < 0.001). (C) Representative images of HE staining in lung nodules of tumor models (magnification ×200, ×400, scale bar 50 μm). (D) Western blot analyzed the protein levels of HMGB1 and SNAI1 in harvested tumor tissues. (E) qRT‐PCR investigated the RSF1‐IT2, miR129‐5p, and SNAI1 expression in harvested tumor tissues (*n* = 3, mean ± SD, *t*‐test, *P < 0.05). (F) Representative images of HMGB1, SNAI1, E‐cadherin immunohistochemical staining with HMGB1, and SNAI1 antibody in LV‐Vector and LV‐HMGB1 groups (magnification ×200, scale bar 50 μm).

## 4 Discussion

HMGB1, as a nonhistone chromosome‐binding protein, could promote tumor invasion and metastasis (Shen *et al.*, 2009; Swartz, 2014). In the present study, we identified HMGB1 expression was significantly increased in NSCLC tissues. HMGB1, a risk factor for death in NSCLC patients, was closely related to advanced TNM stages and poor prognosis. It has been widely studied that extracellular HMGB1 induced tumor progression through binding RAGE and TLRs and then activated its downstream signaling pathways (Angelopoulou *et al.*, 2016; Wang *et al.*, 2015). However, studies regarding the function of intracellular HMGB1 were limited. It was reported that intracellular HMGB1 participated in DNA binding, inhibited apoptosis, enhanced the angiogenesis ability of endothelial cells, and regulated EMT process (Chen *et al.*, 2012; Su and Bi, 2012; Tang *et al.*, 2010b). EMT is one of the initiating factors controlling invasion of epithelial cells (Avtanski *et al.*, 2014; Li and Li, 2015). SNAI1 is a key regulatory factor in the EMT process, which can bind various effector proteins and regulate transcription (Argast *et al.*, 2011; Cheng *et al.*, 2015; Mikami *et al.*, 2011). Our results indicated the EMT markers such as SNAI1, Twist, and Vimentin expression were significantly increased by HMGB1 overexpression. HMGB1 could directly bind the SNAI1 promoter and induce NSCLC invasion through up‐regulating SNAI1 expression. Previous studies demonstrated that SNAI1 was associated with the down‐regulation of E‐cadherin in EMT process (Kroepil *et al.*, 2012). However, our results showed SNAI1 expression increased and E‐cadherin remained unchanged after overexpressing HMGB1. The molecular mechanisms regulating epithelial cohesion in tumor progression were complex. We speculated that HMGB1 affected E‐cadherin expression through other signaling pathways. A previous study indicated HMGB1 made no significant changes in E‐cadherin levels, which may be caused by HMGB1 damaging the epithelial barrier and inducing the distribution anomalies of E‐cadherin (Huang *et al.*, 2016; Wolfson *et al.*, 2011). The damage to epithelial barrier increased macromolecular permeability. E‐cadherin transferred from cell membrane to cell plasma and its expression remained unchanged (Heijink *et al.*, 2010; Wolfson *et al.*, 2011). The relevant mechanisms need to be further developed.

Increasing evidence proved that lncRNAs played vital roles in cancer initiation and progression. Among the differentially expressed lncRNAs, RSF1‐IT2, a newly detected lncRNA, was regulated by HMGB1 and increased the SNAI1 expression in line with our data. Then, how RSF1‐IT2 up‐regulated the expression of SNAI remained to be explored. A previous article proposed a regulatory mechanism in which transcripts could actively communicate to each other through the microRNA response elements (MREs) (Salmena *et al.*, 2011). LncRNA interacted with miRNA acting as ceRNAs to increase the expression of target RNAs, thereby regulating a series of biological behaviors (Cao *et al.*, 2017; Ge *et al.*, 2019). Our data suggested that RSF1‐IT2 could competitively bind miR‐129‐5p and reversely regulate its expression. Thus, we implied that RSF1‐IT2 promoted tumor metastasis through sponging miR‐129‐5p. During our study of how the HMGB1‐RSF1‐IT2‐miR‐129‐5p exerted its influence on lung cancer, an interesting positive loop revealed itself. RSF1‐IT2 overexpression significantly rescued the silencing effect of miR‐129‐5p on SNAI1 protein expression. Moreover, miR‐129‐5p also targeted HMGB1 and regulated EMT process as a tumor suppressor (Li *et al.*, 2017). The above results supported the conclusion that HMGB1 regulated RSF1‐IT2 thus reducing the available miR‐129‐5p to target SNAI1, and HMGB1 was also targeted by miR‐129‐5p in turn, which just formed a positive feedback loop (Fig. 7).

**Fig. 7:** HMGB1 regulates SNAI1 during NSCLC metastasis, through both a direct transcriptional activation and an indirect RSF1‐IT2‐dependent manner.

The lncRNA RSF1‐IT2 was derived from RSF1 gene, and its role in NSCLC had not been reported. RSF1 was highly expressed in various tumors and identified as an independent prognostic marker in prostate cancer (He *et al.*, 2019; Höflmayer *et al.*, 2019). Besides, a previous report analyzed TCGA datasets to systematically identify lncRNAs related to gastric cancer. It was demonstrated that 1294 lncRNAs including RSF1‐IT2 were differentially expressed in gastric cancer. And RSF1‐IT2 was independently associated with overall survival of gastric cancer (Han *et al.*, 2017). On the basis of the above studies, the biological functions of RSF1‐IT2 in NSCLC were further investigated. In our study, RSF1‐IT2 promoted NSCLC cell proliferation and miR‐129‐5p mimics abrogated RSF1‐IT2‐mediated increase in cell proliferation. Collectively, RSF1‐IT2 promoted tumor growth and metastasis at least in part via the miR‐129‐5p axis. Importantly, high expression of RSF1‐IT2 was found closely correlated with tumor progression in both HMGB1‐overexpressed xenograft nude mice and NSCLC patients. These results demonstrated the poorly known RSF1‐IT2 might act as a useful diagnostic biomarker for NSCLC patients.

The present study had confirmed that HMGB1 was a tumor‐promoting factor; however, increasing evidence showed that HMGB1 played dual effects on tumor. On the one hand, HMGB1 could promote the maturation of dendritic cells and enhanced the reactivity to lymph node chemokines, thereby stimulating the occurrence of immune response to produce antitumor effect (Liu *et al.*, 2011). On the other hand, HMGB1 also promoted the tumor angiogenesis thus slowing down the apoptosis of cancer cells (Wu *et al.*, 2018b). Besides, HMGB1 resulted in the resistance of tumor cells to chemoradiotherapy through the release of Beclin1 protein inducing autophagy (Jin and Choi, 2012; Kong *et al.*, 2015). Some studies have shown that the bidirectional effect of HMGB1 on antitumor immunity was closely related to its extracellular concentration and redox status of molecules. High concentration and reductive state of HMGB1 mainly induced autophagy and promoted tumor immune escape, which was related to tumor metastasis (Kusume *et al.*, 2009; Tang *et al.*, 2010a). Further studies are needed to elucidate the mechanism and signaling pathways of HMGB1 and how to activate its own antitumor immunity effect, which will be of great help to the antitumor treatment of HMGB1.

## 5 Conclusions

Our study revealed that HMGB1 enhanced the proliferation, migration, and invasion of NSCLC. We demonstrated that HMGB1 up‐regulated SNAI1 expression in a direct transcriptional activation and RSF1‐IT2‐dependent manner during NSCLC metastasis. RSF1‐IT2 reduced the available miR‐129‐5p to target SNAI1, and HMGB1 was also targeted by miR‐129‐5p in turn. We also firstly reported RSF1‐IT2 played key parts in tumor progression. The findings in this study provided new insights into the understanding of the molecular mechanism involved in tumor metastasis and served a potential prognosis marker and therapeutic target for NSCLC.

## Conflict of interest

The authors declare no conflict of interest.

## Author contributions

XW, YC, and WG performed the experiments and wrote the paper; WG, TL, and HD analyzed and interpreted the data; WW, MX, and GM partially participated in the experiments; XW and DP designed and supervised the project. All authors read and approved the final manuscript.

## Ethics statement

This study was performed under a protocol approved by the Review Board of the Affiliated Xuzhou Municipal Hospital of Xuzhou Medical University, and all examinations were performed after obtaining written informed consents. Animal experiments were in conformance with the Institutional Animal Care and Use Committee of Xuzhou Medical University.

## Supporting information


**Fig. S1.** Heatmap of highly expressed lncRNAs in lung cancer tissues using TCGA database.
**Fig. S2.** qPCR was performed to investigate the lncRNA levels in H1299 cells after transfected with si‐HMGB1 and pcDNA3.1‐HMGB1.
**Fig. S3.** ChIP analysis of RSF1‐IT2 promoter regions used anti‐HMGB1 antibody.
**Fig. S4.** The sub‐cellular localization of RSF1‐IT2.

## Data Availability

The datasets generated during and/or analyzed during the current study are available from the corresponding author upon reasonable request.
